The article "Structural and functional analysis of cases of family treatment treated in the public social services system" was published in 2021. Journal: Heliyon.

# Structural and functional analysis of cases of family treatment treated in the public social services system

**DOI:** 10.1016/j.heliyon.2021.e06825

**Published:** 2021-05-09

**Authors:** Susana Martí-García, Fernando Relinque-Medina, Manuela Ángela Fernández-Borrero, Octavio Vázquez-Aguado

**Affiliations:** a Universidad de Huelva, Huelva, Spain; b Universidad Pablo de Olavide, Seville, Spain; c Research Centre for Contemporary Thought and Innovation for Social Development (COIDESO); d Research Group AGORA – (HU-M648); e Research Group Social Studies and Social Intervention ESEIS – (SEJ-216)

**Keywords:** Family, Situation of risk, Unprotection, Social services, Family Treatment Team, Qualitative method

## Abstract

The purpose of this work has been to analyze, from a structural and functional approach, the families at risk or unprotected by the Family Treatment Teams, inserted in the Public System of Social Services. For this purpose, qualitative research methods and techniques have been used on 26 interdisciplinary reports generated in the most representative cases of family intervention.

Significant results have been obtained describing family structures, life-cycle adaptation, pattern repetition across generations, life events and family functioning, and linked patterns. The data reveal that these are families with common problems related mainly to the behaviour of minors and the coverage of basic needs. Negligence is the central element in this type of families as well as the maladjustment to the life cycle of the family system. All this from patterns of repetition linking dysfunctional.

## 1 Introduction

The family as a social institution, in spite of the historical transformations experienced, continues to be the appropriate context to respond to the evolutionary and developmental needs of people, constituting the ideal environment for child growth and development. For this reason, the domestic context and parental responsibility are increasingly important as primary sources of childcare (López, 2008; Cojocaru and Cojocaru, 2011). However, not all family systems adequately develop their competencies, and they can become contexts of risk or threat to the well-being of children, mainly when there are risk factors that influence the appearance of different forms of child abuse (Fedor, 2011; Rodrigo et al., 2009).

In Spain, the intervention of the Child Protection System was aimed at this type of family, where situations are serious, and measures of helplessness are interposed. From the 1990s onwards, the focus was extended to families at risk, whether of a mild, moderate or serious level. With this, new visions and orientations integrating intervention with aid, support and prevention measures were also incorporated (Casares, 2017).

This article presents the structural and functional analysis of the families’ object of intervention of the provincial Family Treatment Teams inserted in the Child Protection System of Andalusia (Spain)^1^. The components included in the reports of the interdisciplinary team are analyzed. These reports contribute to the professional diagnosis and to the intervention proposals to be developed.

This is an advance in the knowledge of the families with whom these teams work, identifying through a scientific approach their basic structure and functioning. This approach has never been carried out in these regional treatment teams in the region where they perform their professional functions. This analysis will allow the identification of dysfunctional shared elements, as well as key aspects that facilitate the work of these teams from a joint understanding and vision of the reality with which they work.

The approach is carried out from a systemic and ecological conception of the family (Espinal et al., 2006) understanding the holistic nature of its functioning, both of protection elements and of factors associated with risk situations of different levels of gravity. It incorporates analysis of structural components, as well as functional elements related to family dynamics and problems, as well as intrafamily relational patterns and interactions with the environment, in processes of morphogenesis and adaptations.

The Social Services of Andalusia^2^ distinguish two adverse situations in which minors may find themselves within their family nucleus: risk (average level of unprotection) or helplessness (serious level of unprotection). The Programme for the Treatment of Families with Minors at Risk or without Protection^3^ attempts to respond to these family problems within the competence framework of the Child Protection System at the local level, which is where the Family Treatment Teams (here in after, FTT) are located. These are interdisciplinary teams made up of three professionals from the disciplines of Social Work, Psychology and Social Education. These teams develop preventive and protective actions, intervening in an integral way in the family system and, even in its context, if necessary. To this end, it works in coordination with other public systems and social agents, such as the education and health systems or third sector organisations.

The FTT's work through two Subprogrammes: the Risk or Unprotection Subprogramme and the Reunification Subprogramme. The first refers to interventions where there are family situations with deficiencies or difficulties in meeting the needs of minors for optimal development, without requiring the separation of their family system. The Reunification Sub-program is applied at work with those families that have gone through the implementation of a previous protective measure of separation of minors from their family nucleus.

The FTT's have reports made by each professional in the intervention team, as well as an interdisciplinary report. This document is vital in the intervention process, as it provides a complete and joint view of the family situation, as well as a global diagnostic synthesis and assessment and proposals for intevention.

## 2 Literature review

The family is the basic relational unit of society and performs different functions, highlighting those with objectives of an intra-family nature, which pursue the development and protection of members; and others of an extra-family type that seek to accommodate a culture and its transmission.

From the functional and relational perspective, the family is an agent of primary socialization that connects the person to his environment, thus favoring his social integration (Rodrigo and Palacios, 1998). In this sense, the Ecological Theory of Bronfenbrenner (1979), tries to explain the behavior of people putting them in relation with their context, understanding the behavior as a consequence of this interaction. So, the needs and problems related to the daily interaction that a family can present can be of diverse types, among which the following stand out: relational (microsystem) and contextual (exosystem and macrosystem).

From a systemic conception, the family is understood as a system that comprises a set of emotional, intellectual, sentimental situations that are organized in the course of time in several generations (Giberti, 2005). Families may develop in an appropriate manner and in optimal relation to the context or there may be situations in which families may be considered multiproblematic.

For Cancrini (1995, cited in Rodríguez, 2003) the defining characteristics of multi-problem families have to do with the simultaneous presence in two or more members of the same family of structured problematic behaviors, stable in time and serious enough to require external intervention. They count on the existence of serious insufficiency, especially on the part of the parental figures, of the functional and expressive activities necessary to ensure a correct development of family life. In addition, they are characterized by having a chronic relationship of dependence on family support services, and by the development of symptomatic behaviours.

Linares (1997, quoted in Rodríguez, 2003) warns that these multi-problem families should not be seen solely as relational deserts, as there are also compensation mechanisms. When deterioration and disharmony coincide, the ecosystem does not remain passive and sets in motion protective processes that guarantee the continuity of family life, elements that are relevant for family intervention processes.

McGoldrick and Gerson (1985) proposed a categorization of useful elements for analysis and family intervention, factors that have been taken as the object of analysis in this work.

These elements include the family structure, which reflects the composition and configuration of the family system. The adaptation to the life cycle, which can be seen in the adjustment of basic situations of family dynamics. The repetition of patterns across generations, which is about family patterns that are passed down from generation to generation, and it is interesting to note which patterns are the most repeated. For these authors, there are two types of patterns: the symptomatic ones, which have to do with behavioural aspects of one or several members of the system; and the vincular ones, reflected in the different interaction links that are established at the intra-family level. Other elements are the life events and family functioning, which includes the relationship between events in the sphere of individual, family, social, economic and political life, relating them to the impact they have on the family, where a series of general and specific problems are generated in each system as a result of this interconnection. And, finally, the linked and triad patterns that have to do with family relationships. They exist in different forms and characteristics, the most frequent being those of union, fusion, conflict, distancing and rupture. As for the triangles, these authors explain that the family can be understood as a series of interconnected triangulations. They recognize as types of triangles: (1) primary parent with one or more children; (2) perverse, which occurs when there is a coalition between members of different hierarchical levels to attack a third; (3) auxiliary, composed of a single parent, a child and another family member.

In this study, from a systemic conception and reuniting elements of McGoldrick and Gerson (1985), a structural part and a functional part are considered for the analysis, or what Castellón and Ledesma (2012) have denominated as structure and dynamics. The structural part alludes to the elements of family composition, as well as to the presence of situations related to the areas of training, economics, work and the family structure itself. The functional part includes aspects related to transgenerational family dynamics, which includes: adaptation to the life cycle, pattern repetition through generations and life events and family functioning. As well as another dimension that includes relational aspects.

This analysis makes it possible to delve deeper into the family environments in which children and adolescents develop and whose conditions can cause significant damage in the short, medium and/or long term to their well-being and development. Therefore, studying and understanding these realities is essential in order to relate the structure and family events to the social, economic and political context in which they occur. In addition, it allows to know strengths and weaknesses to guide professional decision making.

This study aims to answer questions such as: are there related elements in the family structures of families at risk or unprotected; what are the most present dysfunctional or problematic dynamics; how are the family relationship patterns of the members of the families served by the ETF manifested; among other questions.

It is considered the initial hypothesis of the existence of common structural and functional elements in these families served by the professional teams.

Also, the general objective of this research is to study the structural and functional characteristics of the families subject to intervention for risk or for lack of protection by the Family Treatment Teams of the province of Huelva. The specific aim is, firstly, to ascertain the structural profile of the families served, then to explore the functional dynamics of these families and, finally, to analyse the linked and triangular patterns that have to do with family functioning.

All this will make it possible to highlight the relevance of the information gathered and analysed from professional reports for the preparation of family intervention measures and processes.

## 3 Method

### 3.1 Participants

In this study the object of analysis are the families with minors who have gone through a process of intervention in 13 FTT's. These families have been studied through the Technical Interdisciplinary Report, analyzing a total of 26 family reports, among which 13 from the Risk Subprogram and 13 from the Reunification Subprogram are identified, all of them belonging to the Treatment Program for Families with Minors at Risk or Unprotected. The dates of these reports range from December 2010 to January 2017. These documents have been chosen by each interdisciplinary team as the most representative of their area of focus.

### 3.2 Techniques and instruments

The basic instruments of the analysis are the interdisciplinary reports of the family cases. These reports have a structure composed of the following common elements: (1) data identifying minors; (2) family composition; (3) synthesis and global interdisciplinary diagnostic assessment; and (4) proposal for action to be taken.

### 3.3 Analysis strategy

The methodological strategy used has been qualitative, based on the categorization and codification of the information contained in the reports, and the construction of semantic networks to obtain results and for the development of a theoretical generation. The categories of analysis, supported by the theoretical framework, are those shown in Table 1. Within each of the categories, codes have been assigned that have been the basis for the establishment of semantic networks.

**Table 1:** Categories of analysis.

Structural Characteristics	Functional Characteristics	
	Trans-generational Dynamics	Relationships & Interactions
1. Family structure	2. Adaptation to the life cycle.	5. Relational patterns and triangles
	3 Pattern repetition across generations	
	4. Life events and family functioning	

A combination of inductive and deductive logic has been followed given that, initially, a deductive coding based on theoretically explored categories was carried out in order to carry out an initial systematization of the information.

Later, the analysis was oriented from an open codification and according to an inductive logic. This work is based on Grounded Theory, which is the best way to represent social reality, given that the theoretical explanation emanates from the data (Andréu, García-Nieto and Pérez, 2007). This Theory, although initially prioritizing the inductive approach, contemplates the possibility of establishing a mixed deductive model in the first step, but inductive generating new explanations and theories in the second and last level, granting circularity to the process (San Martín, 2014).

In the process of Theoretical Codification, established the codes, the second process of analysis has determined the belonging of these codes to different theoretical categories, relating categories and subcategories in an axial coding process. Finally, conditional/causal information has been generated, following a selective coding of the most significant nodes based on their density within the network, that is, their relationship with other existing codes in the network. To this end, a hierarchical design network analysis and top-down selection (causes) (consequences) have been carried out, based on top-down logic.

All interdisciplinary reports have been analysed using the qualitative software Atlas.ti version 8. This software has structured the information in a network that has facilitated the semantic structural analysis of the data. It should be noted that there was a saturation of information before the whole process was completed, approximately at the time when half of the reports were analysed.

## 4 Results

The results are presented according to the logic of the proposed objectives. In this order, the most relevant codes can be seen in Table 2.

**Table 2:** Codes by category of analysis from density

Dimension	Codes	Density
Structural Family Characteristics		
1. Family Structure	Vital_Event_Death_Father	7
	Situación laboral_ Desempleo	6
	Single-parent_Family_Type	6
	Vital_Event_New_Partner	5
Functional Family Characteristics		
Transgeneracional		

2. Adaptation to the Life Cycle	Parental_Generalized_Vital_Cycle_Unadaptation	9
	Inadaptation_Vital_Cycle_Parental_Education	5
3.The repetition across generations	Pattern_Repetition_Link_Family_Dysfunction	20
	Pattern_Repetition_Symptomatic_Mental_Health	6
4. Life events and family	Problematic_Behavioral_Minors	17
	Problematic_Basic_Needs_Not_Covered	11
	Problematic_Absence_Consciousness_Problem	10
	Problematic_Economic_Instability	9
	Problematic_Standards/Limits	9
	Problematic_School_Absenteeism	7
	Problematic_Delegitimation_Mother	7
	Problematic_Parental_Implication_Health	7
	Problem_Family_Support_Insufficient	6
	Problematic_Dysfunction_Rol	6
	Problem_Health_Addictions_Drugs/Alcohol	6
	Problematic_Economic_Insufficiency_Resources	5
	Problematic_Housing_Habitability	5

Relationships and interactions		
5. Relational patterns and triangles	Negligence	28
	Domestic_Violence	9
	Gender-Violence	8

From the analysis carried out, a total of 181 codes were obtained, clustered in 23 groups and 64 networks. With the exception of the structural dimension, where descriptive analyses are shown, the rest of the results present those codes and networks that have obtained greater density for each dimension, establishing themselves as the most relevant elements extracted from the discourse. The term density in qualitative analysis refers to the number of relationships that a code has with other codes contained in the discourse.

## 5 Structural family characteristics

The analysis of the network of codes of this dimension has shown that these are families in which those of the reconstituted type stand out as well as those of the single-parent type, the latter formed as a result of a break-up of a couple or the death of the father. The role of care falls mainly on the maternal figure.

Single-parent families are related to temporary work situations. With regard to labour and economic aspects of the rest of the cases, the data show that they are families where unemployment situations or work situations without a contract stand out. To these circumstances are added those of receipt of economic benefits, among which the Non-Contributory Pension^4^ predominates, which is sometimes complemented with work situations without a contract; Family Financial Aid^5^ and the Dependent Child Benefit^6^.

On the other hand, with regard to the training profile, families with primary or intermediate levels of studies are placed.

## 6 Functional aspects of transgenerational dynamics

### 6.1 Family life cycle

In this dimension of analysis, the code of parental maladaptation to the life cycle (density 9) should be highlighted. This code includes all those elements that areframed within the individual and family life cycle. The data reveal that the main causes of this maladjustment come from problems such as parental mental health problem, drug and alcohol addiction of the mother and role dysfunction.

Because of this maladjustment, problematic families associated with the behaviour of minors, the establishment of inappropriate rules and limits by parental figures and the failure to cover the basic needs of minors are generated. It should be pointed out that in the case of single-parent families, the lack of adaptation to the life cycle is usually generated with greater intensity. All this has to do with patterns of repetition linking dysfunctional across family generations.

### 6.2 Pattern repetition across generations

Regarding the repetition of guidelines, it is worth highlighting those of the dysfunctional link type (density 20). This type of link establishes a gear of causes and consequences that are repeated from one generation to the next. It starts fundamentally from causes such as patterns of gender violence, discord or parental and distant or poor relational conflict on the part of parental figures and members of the extended family. Other causes are the absence of parental awareness of the adverse family situation and the delegitimization of the mother. The latter is generally established by the paternal figure since it is associated with situations of gender violence.

These links and problems also generate a pattern of consequences in the families, such as links marked by negligence and domestic violence, as well as behavioural problems of minors and the appropriate constitution of norms and limits. As the data show, the typology of single-parent family is established as a consequence associated with the repetition of linked dysfunctional patterns.

Finally, as has been reflected in the previous point, the consequent maladaptation to the life cycle appear in a generalized way on the part of the parental figures.

### 6.3 Life events and family functioning

According to the results obtained, the most outstanding family problems are related to the behaviour of minors (density 17), the coverage of their basic needs (density 11) and the lack of awareness of family problems on the part of the parental figures (density 10).

As for the behavioural difficulties of minors in the cases analysed, the network reflects causes mainly associated with problems of drug and alcohol addictions accompanied by crimes of actions against public health as well as prison sentences imposed on parental figures and, finally, living in an inadequate context that has a negative influence on this behavioural problem. Linking patterns that generate discord or conflict as well as parental triangulation, which deals with the union between father and mother in relation to the care of a child, are the two types of relationships that most affect as the cause of the behavioral problems of minors.

The consequences of these adverse behaviors affect problems such as the correct establishment of norms and limits, the existence of school absenteeism and the generation of neighborhood complaints. An adverse family system is generated, in which there is domestic violence, and which is framed in a cycle of generalized vital maladjustment with patterns of repetition linked to dysfunctional and symptomatic patterns associated with substance addiction.

With regard to the code that contains quotations on the non-coverage of basic needs, the data reveal that the causes that generate this situation are linked to other difficulties that have to do with parental maladaptation to the life cycle in general, the lack of family and environmental support, the uninhabitability of housing and the insufficiency of economic resources that generate, in addition, economic debts. As for the problems that also affect and have to do with health, those of lack of hygiene and deficient nutrition of minors stand out. Because of these difficulties, a negligent parental bonding pattern is generated, highlighting that the code that collects the typology of single-parent family appears associated as the cause of this problem of coverage of basic needs.

Finally, the lack of awareness on the part of parents of the existence of problems in the system has its main causes in problems that have to do with the mental health of both parents and their lack of interest and collaboration. These circumstances, coupled with this lack of awareness, have as a consequence the appearance of negligent patterns, the repetition of linked patterns of family dysfunction and the chronification of the problem. All these elements lead to a process that ends in the proposal of non-unification by the FTTs.

### 6.4 Functional aspects based on relationships and interactions

Analyses have shown that the relational pattern defined by negligence is the code that has the highest level of importance, being also the one with the highest density of the set of total codes extracted (density 28). In the causes of the hierarchical network, the problems of coverage of basic needs stand out with greater density, as well as the fact that parents are not aware of the existence of problems. Added to this are the codes of insufficient family support and dysfunction of the role of minors, who generally assume adult roles. Finally, another cause to point out is the problem of alcohol addiction of the maternal figure. As for the consequences of these situations of negligence, the most significant code reflects that it is a situation that is repeated in a transgenerational manner, from one generation to the next. In addition, there is the direct consequence of resulting in processes of domestic violence and the difficulty of having rules and limits. The codes of situations of school absenteeism and of problems of parental involvement with professional intervention are also shown as consequences of these situations of negligence.

The domestic violence code (density 9) is significant in this dimension. The main causes of this violence are the existence of previous negligence and repeated dysfunctional relational patterns in families. Other causes are also shown that are less related to other codes, such as the existence of problems related to crimes, the delegitimization of the mother by the father, and perverse triangular relationships. The consequences derive in behavioural problems of minors and in situations of school absenteeism.

Finally, the relationships of gender violence (density 8), rest mainly on causes that have to do with the dependence of the mother to her partner and with patterns of gender violence in other previous relationships of the father. The consequences of this type of violence generated in the family are problematic in the mother of delegitimization, mental health and suicide attempts. It also forms, in a general way, distant patterns of the father with respect to their children. In addition, it is established as one of the causes of couple break-up. This pattern of behavior is associated with the generation of patterns of repetition linking family dysfunction throughout the generations.

## 7 Discussion and conclusions

The families studied are characterized by a series of problems that are common in all cases. On the one hand, it is worth highlighting the position that parental negligence assumes in the results, becoming a central element in the operational structure of the FTTs, and thus be able to respond to the research questions and hypotheses raised.

These are systems in which parents establish intra-family interaction based mainly on the failure to meet the basic needs of their children, one of the most significant consequences in this context being the behavioural problems of minors. All this, generally, is lived from an unconscious look of the situation on the part of the parents, fact that can be related to the relational patterns repetition that are established throughout the generations and that generate in the system situations of apparent normality in actions that really are dysfunctional. Based on this dysfunctionality, families are generated that are in a situation of psychosocial risk (Rodrigo et al., 2008).

These problems are also related to external components such as labour instability and insufficient economic resources. There is no doubt that the economic crisis that has occurred in Spain since 2008 has meant an increase in the need for families to have access to the Public Social Services System and an increase in the complexity of cases, without forgetting the progressive chronification of cases and the situations of dependence on said System generated in the last decade (Garcés, 2012; Laparra and Pérez, 2012). In relation to this, economic protective measures have been established for the family environment, but they have proved insufficient to overcome the state of crisis generated in Spanish households (Navarro, and Clua-Losada, 2012; Lima, 2016). So, these adverse psychosocial circumstances have found their way out in the family itself, fundamentally in its support resources, generating even greater increases in situations of risk or lack of protection in those family systems that, especially if they are single-parent, may lack this type of informal support, as is reflected in the families studied in this work.

On the other hand, the results obtained reveal that patterns of relationships are established across generations that have special to do with situations of domestic and gender-based violence. Two significant problems in the intervention work of the FTTs. It is in this type of interaction that a greater number of triangulations are reflected, although their number has not been significant in the analysis. Domestic violence is a controversial social phenomenon that has recently appeared in family investigations, mainly because of the difficulty of limiting violent behaviour in a private context such as the family. This problem can occur in any of the members of the family nucleus, that is to say, it is a violence carried out within the family by both adults and minors (González, 2012; Fedor, 2011).

With regard to gender-based violence against women, it should be noted that in Spain it has progressively increased, becoming a major social problem.

According to the latest data from the Integral Monitoring System in cases of Gender Violence (VioGén System) (Ministerio del Interior del Gobierno de España, 2018), Spain currently has a total of 476,718 victims, of which 112,358 have been generated in Andalusia, a figure that places this autonomous community at the top of the list in this statistical report. This is also reflected in the reports analyzed, where many of the women who make up these families suffer situations of gender violence.

The analysis carried out in this work highlights the essential and common elements that appear in the cases attended by the ETFs, giving the opportunity to generate changes and/or improvements in professional decision making, thus having direct consequences in the family professional intervention.

The present structure of single parenthood, associated with issues of economic difficulty due to temporary employment and the fact of being a woman (a question of risk and exclusion on many occasions) must be considered as an element of vulnerability from the family intervention. Similarly, public services must take these results into account when planning their interventions. It is a reality that this type of family teams intervene when risk situations have already occurred, but the whole social service system must work not only to repair but also to prevent from the knowledge of these structural, but above all functional, characteristics. Direct results have been extracted related to negligence and issues of addictions and erroneous parental patterns, adding to the lack of awareness of these patterns. Networking, coordinated with education and health systems and services are key to reducing the number of cases that reach these family teams.

It is of vital importance to have at the disposal of these and other professionals’ information on the structure and functionality of the user families, with the aim of carrying out a more effective and efficient work by influencing the situations that constitute the axis of family problems. In this way, the shared economic vulnerability is known, as well as the lack of awareness of how parents themselves act wrongly. However, the context of intervention with families is characterized by focusing their efforts on care and treatment, with aspects such as evaluation and research remaining in the background, despite the existence of some attempts at systematization (Arruabarrena and De Paúl, 2002; Rodríguez et al., 2006).

Conclude by pointing out that the work carried out by these ETFs is fundamental and necessary, even more so if we bear in mind that it is carried out from an interdisciplinary work team. This organization of family intervention acts from an integral, dynamic, adaptive and open plan, in relation, as Hidalgo et al. (2009) say, with the defining characteristics of family systems.

The family constitutes, in a universal way, a social agent and generator of key changes in the individual and social development of people (Escartín, 1992; Rodrigo and Palacios, 1998), this consideration on the part of public organisms should be sufficient to bet, from social policies, on the importance of the protection of the family, childhood and adolescence. All this from a priority and innovative level and of a preventive and promoting rather than palliative and punitive nature (Menéndez et al., 2012).

This study has formed a qualitative analysis that could be extended with a quantitative analysis of the socio-demographic trait of the families served, in order to obtain a more complete picture of the profile of the cases served.

However, this research can serve as a basis for future studies that have to do with family intervention and professional decision-making from public social services, and that guarantee policies and actions based on evidence that can lead to more effective and efficient interventions.

It is important to point out that the study carried out covers a synchronic analysis of 26 families report, this can be a limitation since it shows a reality fixed in time, that can be changing and it would be necessary to extend the study following a diachronic methodology that adapts to the progressive changes of the society in general and of the study group in particular.

It would be interesting to be able to study the comparison of intervention proposals of the different professional profiles that make up the family treatment teams (psychologists, social workers and social educators), as well as to relate their intervention decisions to the type of families or characteristics extracted from this study.

Likewise, according to Huynh (2020), the COVID-19 pandemic situation and the new socio-cultural context that families at social risk must face, open the need for future research to analyse the object of study of this paper in the post-covid era.

## Declarations

### Author contribution statement

Susana Martí-García, Fernando Relinque-Medina, Manuela Ángela Fernández-Borrero, Octavio Vázquez-Aguado: Conceived and designed the experiments; Performed the experiments; Analyzed and interpreted the data; Contributed reagents, materials, analysis tools or data; Wrote the paper.

### Funding statement

This work was supported by 10.13039/501100003176Ministry of Education, Culture and Sport of the Government of Spain through the National University Teacher Training Programme (FPU15/03909).

### Data availability statement

The data that has been used is confidential.

### Declaration of interests statement

The authors declare no conflict of interest.

### Additional information

No additional information is available for this paper.

## Footnotes

1 For information on local Social Services in Spain, please refer to Pastor and Sánchez (2014).

2 Ley 9/2016, de 27 de diciembre, de Servicios Sociales de Andalucía.

3 Regulated and managed by Decree 494/2015, of 1 December.

4 Non-contributory retirement and disability pensions are recognised for persons who have not made sufficient Social Security contributions to obtain a contributory pension.

5 Family Financial Aid is a temporary benefit granted to families with dependent children who are in a vulnerable financial situation that does not cover the basic needs of their children.

6 The Dependent Child Benefit is an economic benefit granted for the birth or inclusion of a new child. The granting of this benefit is subject to special vulnerability cases.

## References

[bib1] Andreu J., García-Nieto A., Pérez A. (2007). Evolución de la Teoría Fundamentada como técnica de análisis cualitativo.

[bib2] Arruabarrena M.I., De Paúl J. (2002). Evaluación de un programa de tratamiento para familias maltratantes y negligentes y familias de alto riesgo. Intervención Psicosocial.

[bib3] Bronfenbrenner U. (1979). Ecology of Human Development: Experiments by Nature and Design.

[bib4] Casares R. (2017). La intervención desarrollada por los equipos de tratamiento familiar. Perfiles familiares atendidos y análisis de la implementación del programa.

[bib5] Castellón S., Ledema E. (2012). *El funcionamiento familiar y su relación con la socialización infantil. Proyecciones para su estudio en una comunidad suburbana de Sancti Spiritus. Cuba.* Contribuciones a las ciencias sociales. http://www.eumed.net/rev/ccss/21/ccla.html.

[bib6] Cojocaru D., Cojocaru S. (2011). The privatization of family and its effects on parenting in Romania. Revista Cercetare şi Intervenţie Socială.

[bib7] Escartín M.J. (1992). Manual de trabajo social (modelos de práctica profesional).

[bib8] Espinal I., Gimeno A., González F. (2006). El enfoque sistémico en los estudios sobre la familia. Revista Internacional de Sistemas.

[bib9] Fedor C.G. (2011). DomesticViolenceonChildren and parental education. Revista Cercetare şi Intervenţie Socială.

[bib10] Garcés A. (2012). Los nuevos retos de los servicios sociales en España.

[bib11] Giberti E. (2005). La familia, a pesar de todo.

[bib12] González M. (2012). Violencia intrafamiliar: características descriptivas, factores de riesgo y propuesta de un plan de intervención.

[bib13] Hidalgo M.V., Menéndez S., Sánchez J., Lorence B., Jiménez L. (2009). La intervención con familias en situación de riesgo psicosocial Aportaciones desde un enfoque psicoeducativo. Apunt. Psicol..

[bib14] Huynh T.L.D. (2020). Does culture matter social distancing under the COVID-19 pandemic?. Saf. Sci..

[bib15] Laparra M., Pérez B. (2012). Crisis y fractura social en Europa. Causas y efectos en España, Colección Estudios Sociales, 35.

[bib16] Lima A.I. (2016). II Informe sobre los Servicios Sociales en España (ISSE).

[bib17] López F. (2008). Las necesidades durante la infancia: una propuesta funcional. En Necesidades en la infancia y en la adolescencia.

[bib18] McGoldrick, Gerson (1985). Genogramas en la evaluación familiar.

[bib19] Menendez S., Arenas A.V., Perez J., Lorence B. (2012). Madres usuarias de servicios de preservación familiar: perfil sociodemográfico y evolución. Cuad. Trab. Soc..

[bib20] Ministerio del Interior del Gobierno de España (2018). Sistema de Seguimiento Integral en los casos de Violencia de Género. http://www.interior.gob.es/documents/642012/8312985/Indicadores+Basicos+Sistema+VioG%C3%A9n+30_11_2018/9eed2f83-8ae2-489e-b583-474d1126f3ca.

[bib21] Navarro V., Clua-Losada M. (2012). El impacto de la crisis en las familias y en la infancia. Observatorio Social de España.

[bib22] Pastor E., Sánchez M. (2014). Analysis and impact of the economic crisis and regulatory changes in the needs and benefits system Municipal social services: analysis case of Murcia-Spain. Revista Cercetare şi Intervenţie Socială.

[bib23] Rodrigo M.J., Cabrera E., Martín J.C., Máiquez M.L. (2009). Las competencias parentales en contextos de riesgo psicosocial. Psychosoc. Interv..

[bib24] Rodrigo M.J., Máiquez M.L., Martín J.C., Byrne S. (2008). Preservación familiar. Un enfoque positivo para la intervención con familias.

[bib25] Rodrigo M.J., Palacios J. (1998). Familia Y Desarrollo Humano.

[bib26] Rodríguez M. (2003). La familia multiproblemática y el modelo sistémico. Portularia.

[bib27] Rodríguez G., Camacho J., Rodrigo M.J., Martín J.C., Máiquez M.L. (2006). Evaluación de riesgo psicosocial en familias usuarias de servicios sociales municipales. Psicothema.

[bib28] San Martín D. (2014). Teoría fundamentada y Atlas.ti: recursos metodológicos para la investigación educativa. Rev. Electrón. Invest. Educ..

